This article has been retracted.

# Value of ddPCR in the Preoperative Diagnosis of Solitary Pulmonary Nodules Based on the Observation of Virtual Reality Images of Smart Medical Treatment

**DOI:** 10.1155/2021/9920617

**Published:** 2021-08-12

**Authors:** Xuri Mou, Guiying Sun, Yubo Shi, Liangdong Zhang, Runjie Li, Shuling Yu, Shuliang Liu

**Affiliations:** Department of Chest Surgery, Yantaishan Hospital, Yantai 264000, Shandong, China

## Abstract

At present, lung cancer ranks the first cause of tumor death in the world, and malignant tumors in the SPN detected by imaging account for 5–40%, most of which are peripheral lung cancer. The recovery of the solitary nodules in the lung after treatment has also been paid attention to. In order to explore the correlation of solitary pulmonary nodule (SPN) with microvessel density (MVD), vascular parameters, and vascular ratio under virtual reality images of smart medical treatment and evaluate the differentiation of SPN by ddPCR under virtual reality image observation diagnosis value, this article collects relevant information by investigating patients, investigating relevant literature, interviewing professionals, and constructing a case template, using a comprehensive quantitative and qualitative analysis method to create a damage assessment matrix. Experimental results prove that there are significant differences in the microvascular architecture within the SPN in the benign, inflammatory, and malignant groups. The correlation between ddPCR and vascular parameters (especially the ratio of luminal vessels) under the virtual reality image observation of smart medical treatment is better than other detection methods, and its accuracy is about 10% higher. Based on the observation of smart medical virtual reality images, ddPCR can be used as an index for noninvasive evaluation of tumor angiogenesis, which is helpful for the differential diagnosis of SPN.

## 1. Introduction

SPN refers to a single circular oedema with a diameter of thirty kilometres in the pulmonary spine, with clean edges, without loss of control, satellite damage, and enlargement of the median ganglia. It is a common clinical lung disease [1]. Currently, lung cancer ranks as the first cause of death from a tumor in the world, and the malignant tumors in the SPN were detected by imaging for 5–40%, most of which are peripheral lung cancer. The five-year survival rate after the surgical dissection of early lung cancer may be as high as 54–73%, while the rate of advanced lung cancer is only 2%. Therefore, early diagnosis and treatment of solitary pulmonary oedema cannot only improve the therapeutic effect of malignant tumors and improve prognosis, but also avoid the physical and financial burden caused by excessive treatment of benign harm [2]. Today, SPN therapy emphasizes early detection, early diagnosis, early treatment, and early recovery to improve the prognosis and reduce the degree of injury to patients.

With continued advances in science and technology, medical imaging technology has developed rapidly, and a large number of advanced medical imaging facilities such as CT (computational tomography) and MR (nuclear magnetic resonance) have appeared in a short period of time [3]. The continuous improvement of computer processing capacity and the rapid development of modern technology information provide the necessary conditions for the display of virtual reality imaging technology. Virtual endoscopy is a special three-dimensional visualization tool. With the help of computer software, it can create the interconnectedness of the anatomical structure. This imaging tool can obtain images similar to the traditional endoscope, but it is a noninvasive way compared to the traditional endoscope [4–6].

Maki believes that, in recent years, patient specific CT/MRI data have been used as clinical XR (extended reality) by medical image analysis, including virtual reality (VR), augmented reality (AR), and hybrid reality (MR), for planning and simulating treatment procedures, navigation, and training. Clinical XR applications can be built using cheap 3D reconstruction software and web services. The key to develop this technology is to extract organs automatically through artificial intelligence and deep learning [7]. Li believes that neuroanatomy is complex and difficult to master. The operation is difficult and requires a high level of minimally invasive refinement. In addition, the teaching, training, and anatomy methods of neurosurgery are also limited. At present, the application of virtual reality technology in neurosurgery teaching and clinical practice has been reported, but the application of augmented reality technology in neurosurgery teaching is rarely reported. It introduces the multimodal neural navigation planning platform and analyzes and discusses the application of virtual reality and augmented reality technology in neurosurgery teaching [8]. Geetha reviewed the development of virtual reality (VR) and augmented reality (AR) in recent years, from the beginning of dental history to the progress of dental technology. Due to the lack of technology, we need to rely on other instruments to improve the success rate of surgery and reduce the risk of surgery. The development of tracking devices has changed the way of surgery and education. Clinical surgery is based on mature education. Virtual reality and augmented reality affect the skills of training courses and navigation system at the same time. Virtual reality and augmented reality technologies not only are widely used in dental training courses and surgery, but also improve people's lives in various fields [9]. Fang believes that smart medicine can provide two types of feedback for patients receiving rehabilitation training. This is the biggest advantage of virtual reality technology for rehabilitation training, and it can improve patients' perception of rehabilitation effect. This paper studies the application of virtual reality technology in the practical teaching of sports rehabilitation major. This paper adopts the research method of virtual scene location mapping. Virtual scene position mapping is a virtual implementation technology based on upper limb rehabilitation training, which is operated by the movement of patients' upper limbs. In this experiment, the first- and second-year students of physical rehabilitation major in a local university were tested theoretically and evaluated practically. The experimental data show that the excellent rate and passing rate of practical ability test in the experimental class are significantly higher than those in the control class [10].

This study introduces the microvessel density and the parameters of luminal vessels, namely, the number of luminal vessels, the area of luminal vessels, and the circumference of luminal vessels to quantitatively analyze the microvascular composition of SPN and compare and analyze its correlation with CTPI parameters of nodules, in order to study SPN of different natures. CTPI features provide more objective theoretical support, thus improving the diagnosis and differential diagnosis of SPN. In different clinical studies, researchers have provided us with a variety of risk factors related to lung cancer. These factors include the patient's behavior, genetics, and some inherent characteristics of the patient. They provide us with the opportunity to study the imaging characteristics of different SPNs. It provides a more objective theoretical basis.

## 2. Preoperative Auxiliary Methods for Solitary Nodules in the Lung

### 2.1. Smart Medical

With the rapid development of digital healthcare, electronic health data have grown exponentially [11, 12]. The way in which enormous medical and health data are used to improve the level and quality of medical and health services is one of the current hot issues under investigation. Medical care is closely linked to the life of users [1, 13]. Excellent service design can optimize users' medical procedures, improve users' medical experience, and provide users with better services. The purpose of the self-service system for medical services is to create a convenient, intelligent, standardized, reliable, and open medical service for the environment. Effective use of medical resources helps to solve the problem of long queues for registration in hospitals with “three longs and one short,” long queues for treatment, long queues for payment, and short treatment time. Breaking the traditional way of seeking medical care and creating a new way of seeking medical care, self-service users can complete medical services such as registration, payment, special appointment numbers, laboratory examination printing, and drug withdrawal at the end of the medical service, which not only saves users time, but also improves the efficiency of the process. It saves the hospital's human resources and enables the hospital to adjust resources more reasonably [14]. Simplified medical procedures enable the normal operation of the hospital, which can receive more patients and benefit the society [15].

The medical service system based on the perspective of smart medical care enables hospitals not only to provide users with medical services, but also to provide more detailed services, such as health management, disease prevention, and creating health files for users [16, 17]. Selecting a topic introduces the idea and method of the “Service Design Observation Experience Process for the first time user +, including all + specifically for” creation of a perfect user experience. When designing an intelligent medical system, the service system is designed by analyzing user needs and key touch points, and a comprehensive survey of medical procedures and user experience is carried out to form a system network of doctor-Internet + medical experience [18].

The main development objective of smart medicine is the application of technology and operation. In the current medical environment, how to better understand and transform user expectations and needs and how to use virtual reality technology to better integrate product structure and functions with user needs are key issues in clinical medicine [19, 20]. The key points of the application conform to the following formula:

(1) $$\begin{array}{c} M=\frac{x}{\left(x+i+1\right)},\\ P_{LA}=L_{A}+\left[\frac{D_{A}-\left(L_{A}+1\right)}{C_{\text{skip}}\left(d\right)}\right]\times C_{\text{skip}}\left(d\right)+1,\\ d\left(x_{i},x_{j}\right)=\sqrt{\left({\left|x_{i1}-x_{j1}\right|}^{2}+{\left|x_{i2}-x_{j2}\right|}^{2}+\cdots +{\left|x_{in}-x_{jn}\right|}^{2}\right)}. \end{array}$$

According to the characteristics of the medical system, we have improved the relevant calculation functions:

(2) $$\begin{array}{c} f\left(i\right)=x_{0}+x_{1}y_{1}+x_{2}y_{2}+x_{3}y_{3},\\ W=\frac{N_{1}r_{1}^{2}}{2}+\frac{N_{2}r_{2}^{2}}{2}+N_{2}d_{2}^{2}+\left(\frac{N_{3}r_{3}^{2}}{2}+N_{3}d_{3}^{2}\right)*0.1+\frac{2}{3}N. \end{array}$$

### 2.2. Virtual Reality Technology

Virtual reality technology is an interactive dynamic virtual environment constructed through sensor technology, computer, and artificial intelligence that can act on human perception, making people seem to be in it [21]. Virtual practice is the product of the rapid development of computers, the Internet, information technology, and virtual reality technology. This type of practice is separated from scientific practice and forms a new practice mode. The usual virtual practice refers to the purposeful and two-way object-oriented perceptual activities of the subject in the virtual environment through digital media [22]. Unlike traditional practice, virtual practice has the characteristics of interaction in real time, virtual reality, and the deepening of communication. Its practice process is not restricted by external objective conditions, transcends the limitations of time and space, and can act on objective reality (Figure 1).

Virtual endoscopy is the perfect combination of computer technology and modern medicine. It uses medical equipment to get the original image, which combines many types of IT technologies resulting from the successful application of imaging technology [23]. The greatest improvement in virtual endoscopy and traditional optical endoscopy is that it does not need to enter the human body and does not cause injury to the patient. It is a completely painless method of examination, used for medical diagnosis, surgical planning, and training methods for medical staff [24].

Technology is an instrumental means created by mankind in order to better achieve practical goals in the process of practice [25]. Since ancient times, the development of technology has always evolved under the trend of human pursuit of convenience, simplicity, and efficiency. And “virtual” is a philosophical category that marks freedom and transcendence and embodies the way of thinking and practice that transcends reality [26]. From the trend of technological development, a kind of virtuality that transcends reality and nature is always running through it. For a long time, human beings have been full of curiosity about the unknown world and fantasy creation, so cultural symbols such as religion have been created, the prophecy and mythology of civilization. However, communication methods such as mere words, symbols, and language are restricted by technology, have great limitations in practice and cognitive activities, and cannot give people an immersive communication experience. Therefore, this kind of virtuality has an experience effect that people have been trying to achieve [27].

(3) $$\begin{array}{c} q=\beta *\partial *\left[{\left(\frac{t_{1}}{100}\right)}^{4}-{\left(\frac{t_{2}}{100}\right)}^{4}\right],\\ Q=\frac{\gamma }{t}A_{n}\left(T_{m}-T_{n}\right). \end{array}$$

It can be foreseen that the application fields of virtual reality technology are more extensive than virtual practice. In addition to meeting people's intuitive requirements for face-to-face communication when socializing, it can also use its superior characteristics to break through the constraints of time and space and physical conditions [28]. Its practical activities can also be applied to industry, aerospace, education, retail, and entertainment [29]. In addition, virtual reality technology is also reconstructing the way of thinking of the subject of practice, reshaping people's social relationships, and enriching human spiritual products. Virtual reality practice is bound to become an important turning point in the development of human practice activities [30].

Virtual reality technology is different from traditional media. In a virtual information environment, the user is not only an information publisher, but also a means of dissemination and, at the same time, a receiver of information. This kind of media technology itself is an information field. There is no information centre or authority in this field. Every entrance of virtual reality is the receiver, relay, or sender of information [31]. When we are in virtual reality, we may be confronted with a “dehumanized” virtual object. Perhaps this object is an object shaped by the subject's consciousness, but we can communicate with it like a stranger. On a level, we are our own communication, but the object is a substantive ideal object in our own imagination. But unlike the split personality, under the technology of artificial intelligence, the object we conceive can become a dual existence with both self-consciousness and characteristics endowed by the subject. In this communication process, media technology not only creates the subject, but also acts as an intermediary and also acts as a receiver of the object. This trinity brand-new communication method did not exist before the maturity of virtual reality technology [32].

### 2.3. Droplet Digital PCR

Real-time fluorescent quantitative PCR is widely used in the quantitative detection of viruses. It has the advantages of simple operation, high sensitivity, strong professionalism, fast speed, and high performance [26]. However, RT-qPCR should be based on a standard quantitative curve. The quality of the standard curve is sensitive to factors such as the initial concentration and the concentration of the detector. The purity of the DNA does not match the standard, resulting in its accuracy not meeting the requirements of absolute quantification [33]. In addition, RT-qPCR is sensitive to the effects of reaction inhibitors and is prone to false negatives, which affects the judgment of the results.

The droplet digital PCR (ddPCR) method is a new technology, the detection method is fast and accurate, and it can achieve absolute quantification. Unlike the traditional RT-qPCR method, it is not based on a standard curve, and the quantitative results are more accurate. The ddPCR method is based on serially diluting the sample at a specific concentration and assigning it to a certain number of droplets. Therefore, the number of standards in most droplets is 1 or 0, and then each droplet is treated as an independent auxiliary unit performing PCR [34]. After completing the assistance, the fluorescence signal should be read in each drop. According to the Poisson probability distribution function, the number of original DNA copies in the sample can be calculated [35]. This method uses endpoint detection and is not based on the Cq value. Therefore, the effectiveness of the ddPCR is significantly reduced due to aid, which improves the tolerance of reaction inhibitors and improves the accuracy and repeatability of the method [36, 37].

We use the entropy weight method to determine the weight of each attribute [38].

(4) $$\begin{array}{c} t=\frac{1}{\ln\;x}\sum_{n=1}^{1}f_{nm}*\;\ln\;f_{nm},\\ r=\frac{1-\sum_{n=1}^{x}z_{nm}}{y-\sum_{m=1}^{m}t}. \end{array}$$

Among them

(5) $$\begin{array}{c} f_{mn}=\frac{z_{nm\left(r_{nm}-uq_{m}\right)}}{\sum_{n=1}^{x}z_{nm}},\\ \sum_{m=1}^{x}w_{m}=1. \end{array}$$

Set objective weights for each user attribute:

(6) $$\begin{array}{c} d=\sqrt{\sum_{m=1}^{x}w_{n}*{\left(r_{nm}-uq_{m}\right)}^{2}},\\ w_{n}=\frac{1}{1+d\left(r_{n},uq\right)}. \end{array}$$

From this, the matching value *Q* can be obtained:

(7) $$\begin{array}{c} Q_{\delta }=\left\{r_{n}\left|d\;\cos\left(r_{n},uq\right)\right|\geq \delta \right\}, \end{array}$$

Recognition degree under computing resources

(8) $$\begin{array}{c} \cos\;m\left(r,uq\right)=\alpha *\;\cos\left(r,uq\right)+\left(1-\alpha \right)*\frac{1}{m}\sum_{n=1}^{m}\delta_{ij}. \end{array}$$

The simulation parameters are calculated as follows:

(9) $$\begin{array}{c} F=\frac{\sum \left(q_{rp,rpn}-q_{rpm}\right)\left(q_{uq,uqn}-q_{uq}\right)}{\sum_{n=1}^{n}\left(q_{r}-q_{uq}\right)\sqrt{\sum {\left(q_{uq,uqm}-q_{uq}\right)}^{2}}}. \end{array}$$

Use digital QX100 drop PCR system D level (including droplet production board, droplet generator, PCR machine, and droplet analyzer) for experiments. The experimental steps of digital PCR droplets should include system preparation, droplet production, amplification cycle, and signal reading. ddPCR uses the same initiator and detector as RT-qPCR. The entire ddPCR system is 20 mL, of which 10 mL 2-xddPCRSupermixD is 0.9 mL for the probe, the air star and the lower star (900 nmol/L) each are 0.9 mL, the detector (250 nmol/L) is 0.5 mL, and the DNA standard is 2.5 mL. To generate droplets, use the corresponding droplet creation card and droplet generator, add 20 mm PCR system and 70 mm droplet oil to the droplet generation card, cover with special rubber, and put the raw materials into the droplet generator; the generated droplets are transported to the 96 brake disc and placed in the PCR machine for support. The aid procedure is as follows: 95 : 10 minutes, 95–8451 s, 10 seconds, 58–8451 s, 60 seconds, a total of 40 cycles; after the end of the aid, heat inactivation was in 98–8451 s for 10 minutes. Each template has three repetitions. After reinforcement, the 96-axis plate was placed on the droplet reader to read the signal [39], and Quanta Soft software was used for data analysis.

After treatment, some patients only rely on subjective feelings, and some patients may be afraid of taking the drug for a long time so causing adverse events, usually in a short period of time, or the blood lipids return to the “normal range” and then start to stop the drug. However, the therapeutic drug has many effects, not a simple lipid-lowering drug. It has an important role in stabilizing plaque, improving vascular endothelial function and antiatherosclerosis. As medical staff, in the process of preventive medication for patients, the patient's own economic situation should be fully considered. When the economic level allows, patients should be advised taking drugs with higher cost-effectiveness and efficacy as much as possible, and patients should be encouraged to take long-term medications to improve medication compliance shortening the distance between clinical practice and prevention guidelines.

## 3. Preoperative Auxiliary Experiment for Solitary Pulmonary Nodules

### 3.1. Subjects

Take the patients with SPN problems in the lungs of hospitals in this city as the experimental subjects, collect their clinical data (gender, age at diagnosis or diagnosis, clinical symptoms and signs at admission, auxiliary examinations, etc.), and follow up by telephone consultation and outpatient visits.

Case inclusion criteria are as follows: ① SPN was found on chest CT and surgical resection was performed in advance. ② Dual-source CT perfusion scan was successfully performed on SPN before operation. ③ No antitumor therapy (radiotherapy, chemotherapy, etc.) was performed before surgery. ④ The time of CT perfusion scan is no more than 2 weeks from the operation time.

Case exclusion criteria are as follows: ① the SPN diameter being less than 10 mm; ② patients whose calcification and necrosis area in SPN are too large to measure perfusion data; ③ having a history of iodine contrast agent allergy, ④ being pregnant, parturient, and lactating women; ⑤ patients with severe heart, lung, and kidney insufficiency; and ⑥ unsatisfactory pathology and perfusion image quality.

### 3.2. Image Processing

After receiving the reconstructed image, apply perfusion-related software for postprocessing. Select the tumor program and go through the steps of motion correction (dynamic correction), segmentation (threshold selection), vessels (select reference blood vessel), and other steps to obtain the T-DC curve and perfusion parameters of the lesion area (BV, BF, PMB, MTT, etc.). The mathematical model is a deconvolution method. Select the reference vessel and draw the region of interest (region of interest, ROI): conventionally select the thoracic aorta as the reference vessel, and if the artery is not within the lesion range, select the common carotid artery or the brachiocephalic trunk. Place the ROI at the largest level of the SPN and manually outline the ROI area as much as possible to be consistent with the outer edge of the lesion. The distance between the *X*, *Y*, and *Z* axis tumors should not be less than 2-3 mm as the standard, while avoiding the necrosis, hemorrhage, calcification, and calcification of the tumor. Finally, two experienced imaging physicians measured the SPN perfusion parameter values separately under the double-blind method. If the difference between the two results is greater than 10%, the measurement is repeated once and the average value of the four results is finally taken.

### 3.3. Baseline Data

1. Data content: general information of patients, such as age, gender, ISS score, cause of injury, total operation time, recovery time, intraoperative blood loss, hospitalization time, and complications, was collected.
2. Methods: the electronic medical record system of the first hospital in our city was inquired. According to the clinical diagnosis of patients and the above screening criteria, the qualified patients' information was found. The patients' medical records were borrowed in the medical record room to view the relevant information of patients and collect the relevant information of patients.

### 3.4. Statistics

All data analyses in this article use SPSS19.0, statistical tests use a two-sided test, the significance is defined as 0.05, and *P* < 0.05 is considered important. The statistical results are presented as the average deviation (x.SD). When the test data correspond to the normal distribution, the double *T* test is used for intragroup comparison and the independent *T* sample test is used for intergroup comparison. If the regular distribution is not sufficient, two independent samples and two relevant samples shall be used for inspection.

## 4. Preoperative Auxiliary Experimental Study of Solitary Pulmonary Nodules

### 4.1. Patient Situation

Through hospital admission records, we have collected statistics on patients who have received ischemic stroke in the hospital and classified them according to the cause of their stroke, as shown in Table 1.

From Figure 2 we can see that the overall number of SPNs has shown an upward trend year by year. From 2011 to 2020, the overall number of patients has increased by about 20%. Tuberculosis is an important factor leading to SPN, which causes the proportion of SPN to increase. The increase from 20% in 2010 to about 25% in 2020 needs to arouse people's attention. We classify the severity of SPN in patients, as shown in Table 2.

From Figure 3, we can see that aspergillosis is extremely harmful in SPN, and its proportion of patients far exceeds other causes of SPN, accounting for more than 30% of the total number of patients. This shows that SPN is induced by aspergillosis. The possibility is much higher than other factors. In the case of preventing the occurrence of SPN, special attention should be paid to the impact of aspergillosis.

### 4.2. Different Degrees of SPN Image Differences

We examine different patients and count the various parameters of the patients to check the severity of the patients' SPN, which is divided into three categories: benign, malignant, and inflammatory. The classification parameters are shown in Table 3.

As shown in Table 3, we use BF, BV, and other parameters to classify SPN patients into three groups: benign, inflammatory, and malignant. From the table, we can clearly see that there are obvious differences in the parameters of different types of patients, benign and malignant. The difference between the BF values is about 60. It can be clearly seen from the graph that we display different types of SPN images, as shown in Figures 4–6.

As shown in the figures, there are obvious differences in the image display of patients with different degrees of SPN. The lungs of benign and nauseous patients are clearly different. The BF and BV images between the two are obviously inconsistent and can be easily distinguished. And in the values of SMA and CD34, there are very obvious differences in the imaging of patients at various levels.

### 4.3. Preoperative Auxiliary Effect

We make statistics on the treatment effect of SPN patients and use the calculation model to make the effect numerical and convenient statistics, so that the comparison of treatment effect is more obvious. The specific results are shown in Table 4.

From Figure 7 we can see that, compared to other methods, not only ddPCR therapy based on visual imaging of virtual reality can remain stable during the processing process, but also the data are better than other treatment methods, and the effect is 10% higher. Its performance in other aspects is also very good. For patients with SPN, prudence is extremely important. In this context, we have measured several important indicators of preaccession assistance, which are listed in Table 5.

As shown in Figure 8, in terms of prognosis, the use of ddPCR for the treatment of SPN also has many advantages in preoperative secondary therapy, and its rating is basically above good. Although other methods have their own advantages, in general, ddPCR can play an important role in the prevention of AIDS.

## 5. Conclusion

SPN is the difficulty and focus of chest imaging diagnosis. ddPCR is one of the effective measures to improve the ability of predicting SPN and correctly explain the characteristics of solitary pulmonary nodules as soon as possible. The ddPCR result under the virtual reality image is not “1 + 1 = 2,” but “1 + 1 > 2.” Combining the morphological characteristics of high-resolution CT and the FDG metabolic characteristics provided by PET, the diagnosis is accurate and has further guiding significance. We can know that it is used to predict benign and malignant SPN. This method has the characteristics of high diagnostic accuracy, simplicity, and practicality and is not only suitable for imaging diagnosis but also for clinical treatment. Most of the existing SPN mathematical models are based on the characteristics of the migrant population, and most of the domestically produced models are based on the migrant population to study the morphological characteristics of SPN, that is, the benign and malignant model for predicting SPN based on CT performance and the metabolic characteristics of RET. This study also has some shortcomings. For example, although various measures are being taken to reduce the X-ray dose, the patient will still receive a certain amount of it. The number of experimental cases is relatively small, the nature of SPN is different, and the ratio of inflammatory SPN to benign SPN is also very different. There are sample differences that may affect the stability of the results. Further investigation is needed to increase the number of cases of inflammation and benign diseases. Therefore, in order to evaluate the description of SPN more completely and accurately, a description method is not enough. Seeking a common characterization of multiple models and technologies will become an important development trend.

## Figures and Tables

**Figure 1:** Application of virtual reality technology in medical treatment (from https://image.baidu.com).

**Figure 2:** The cause of the patient.

**Figure 3:** The proportion of patients with SPN degree.

**Figure 4:** Benign SPN display (from https://image.baidu.com). (a) Patient's lung window scan, (b) BF perfusion pseudocolor map, (c) BV perfusion pseudocolor map, (d) SMA immunohistochemistry map, and (e) CD34 immunohistochemistry map.

**Figure 5:** Malignant SPN patient display (from https://image.baidu.com). (a) Patient's lung window scan, (b) BF perfusion pseudocolor map, (c) BV perfusion pseudocolor map, (d) SMA immunohistochemistry map, and (e) CD34 immunohistochemistry map.

**Figure 6:** Image display of patients with inflammatory SPN. (a) Patient's lung window scan, (b) BF perfusion pseudocolor map, (c) BV perfusion pseudocolor map, (d) SMA immunohistochemistry map, and (e) CD34 immunohistochemistry map.

**Figure 7:** Comparison of SPN treatment effect.

**Figure 8:** Changes in prognostic data.

**Table 1:** Causes of stroke over the years.

Causes	2011	2012	2013	2014	2015	2016	2017	2018	2019	2020
Tuberculosis	28	24	20	18	23	13	16	12	17	22
Inflammatory myofibroblastoma	22	19	21	15	20	28	13	20	23	25
Aspergillosis	15	11	18	19	24	18	14	21	20	22
Large cell neuroendocrine carcinoma	16	19	20	16	11	20	25	17	22	21
Small cell carcinoma	23	17	19	21	13	18	19	23	21	15
Alveolar cell carcinoma	20	18	21	23	16	20	19	22	18	19

**Table 2:** Degree of SPN of patients.

	Tuberculosis	Inflammatory myofibroblastoma	Aspergillosis	Large cell neuroendocrine carcinoma	Small cell carcinoma	Alveolar cell carcinoma
Benign	48	24	30	18	23	18
Inflammatory	12	19	9	13	17	21
Malignant	22	17	18	21	9	12
Unknown	15	7	16	11	7	9

**Table 3:** Patient SPN classification.

	Benign group	Inflammatory group	Malignant group	*P*
BF	36.88 ± 3.77	78.56 ± 8.23	97.35 ± 5.78	*P* < 0.05
BV	5.69 ± 4.32	8.79 ± 3.58	11.23 ± 4.85	*P* < 0.05
MTT	12.34 ± 5.81	7.56 ± 4.25	6.48 ± 3.45	*P* < 0.05
SMA	9.24 ± 3.52	13.52 ± 4.72	23.89 ± 5.32	*P* < 0.05
CD34	4.25 ± 2.35	9.25 ± 3.14	12.47 ± 4.91	*P* < 0.05

**Table 4:** Effects of different treatment methods.

	Inflammatory myofibroblastoma	Aspergillosis	Large cell neuroendocrine carcinoma	Small cell carcinoma	Alveolar cell carcinoma
Virtual reality technology	0.537	0.887	0.528	0.718	0.642
Anticoagulant therapy	0.431	0.573	0.431	0.752	0.669
Platelet aggregation therapy	0.479	0.526	0.888	0.697	0.477
Augmented reality technology	0.539	0.643	0.542	0.573	0.681
ddPCR	0.879	0.735	0.779	0.727	0.813

**Table 5:** Prognostic effects.

	Stability	Flexibility	Cerebral infarction	Recovery effect	Pain	Sequelae
Virtual reality technology	0.478	0.817	0.559	0.697	0.679	0.542
Anticoagulant therapy	0.431	0.573	0.431	0.752	0.669	0.678
Lung recovery effect	0.479	0.526	0.823	0.697	0.435	0.617
Augmented reality technology	0.539	0.643	0.556	0.573	0.681	0.554
ddPCR	0.842	0.798	0.697	0.735	0.506	0.489

## Data Availability

Data sharing is not applicable to this article as no datasets were generated or analysed during the current study.
